This article has been retracted.

# Growth inhibition and apoptosis induced by 6-fluoro-3-formylchromone in hepatocellular carcinoma

**DOI:** 10.1186/1471-230X-14-62

**Published:** 2014-04-03

**Authors:** Yijie Zhang, Kailian Zheng, Hongli Yan, Gang Jin, Chenghao Shao, Xuyu Zhou, Yingqi Zhou, Tianlin He

**Affiliations:** 1 Department of General Surgery, Changhai Hospital, No.168 Changhai Road, Shanghai, Yangpu District 200433, China

**Keywords:** FCC, Cell Proliferation, Apoptosis

## Abstract

**Background:**

Hepatocellular carcinoma (HCC) is one of the most lethal and prevalent cancers in human population. The 6-fluoro-3-formylchromone (FCC) has been shown to have anti-tumor activity against various tumor cells. However, the effects of FCC on HCC cell lines have not yet been reported. This study aims to research the effects of FCC on HCC and advance the understanding of the molecular mechanism.

**Methods:**

HCC cell line SMMC-7721 was treated with FCC at various concentrations (0, 2, 5, 10, and 20 μg/ml) for 24, 48 and 72 h, respectively. The proliferations of SMMC-7721 cells were measured by MTT assays. After cultured 24 hours, cell cycle distribution and apoptosis were determined by flow cytometry. However, the expression levels of PCNA, Bax and Bcl-2 were measured by western blotting after 48 hours.

**Results:**

FCC displayed a dose- and time-dependent inhibition of the SMMC-7721 cell proliferations in vitro. It also induced apoptosis with 45.4% and caused cell accumulation in G0/G1 phase with 21.5%. PCNA and Bcl-2 expression was significantly suppressed by FCC in a dose-dependent manner (P < 0.05), while Bax expression was increased.

**Conclusions:**

FCC could significantly inhibit HCC cell growth in vitro through cell cycle arrest and inducing apoptosis by suppressing PCNA expression and modulating the Bax/Bcl-2 ratio.

## Background

Hepatocellular carcinoma (HCC) is the fifth most common cancer and the third common cause of cancer death in the human population [1-4]. HCC is typically aggressive and intrinsically resistant to conventional therapies such as radiotherapy and chemotherapy [5-7]. Therefore, more effective therapeutic agents for treating HCC are desirable.

Previous studies have shown that chromone can induce apoptosis of tumor cells and inhibit tumor growth both in vitro and vivo [8,9]. The derivatives also showed promising activity against various cancers such as pancreatic, prostate, breast, adenocarcinoma and non-small cell lung carcinoma cancers. They can affect multiple signaling pathways, such as NF-ĸB and PI3K/Akt pathways, which play important roles in mechanism of carcinogenesis [10-12].

In eukaryotic cells, PCNA plays a crucial role in DNA replication, repair and cell proliferation in HCC [13]. This protein was involved in synthesis of lead- and lag- DNA strands and provided an anchorage site [14]. Applied inhibitor to down-regulate PCNA expression may cause the cell growth inhibition. Moreover, Bcl-2 family of proteins showed the regulation function of mitochondrial-mediated apoptosis [15]. In addition, Bcl-2 family are classified into two opposing subfamilies, and Bcl-2 and Bax are the most representative members, respectively [16].

3-formylchrome, one of chromone derivatives, shows significant tumor-specific cytotoxicity, dose-dependently induced apoptosis in human oral squamous cell carcinoma cell line (HSC) and human promyelocytic leukemia cell line (HL-60) [17]. It is also reported that some 3-formylchromone derivatives represent more potent cytotoxic activities against some tumor cells but low cytotoxicity against normal cells [18,19]. Among these 3-formylchromone derivatives, 6-fluoro-3-formylchromone (FCC) was proved to be a modifier of multidrug resistance in mouse lymphoma cells and in human Colo320 colon cancer cells [18]. Moreover, Kawase et al. have confirmed that FCC is one of the most cytotoxic 3-formylchromone derivatives against tumor cell lines, such as HSC-2, HSC-3, HL-60 and human submandibular gland carcinoma cell line, through the experiments which described the effects produced by 3-formaychromones replaced at the C-6 position and evaluated the cytotoxicity against various human cell lines [19]. Meanwhile, normal cells of human gingival fibroblast (HGF), human pulp cell (HPC) and human periodontal ligament fibroblast (HPLF) exhibit a higher immunity to FCC as compared with the tumor cell lines [19]. FCC is a promising approach for tumor treatments. Nevertheless, to the best of our knowledge, there is little report describing the effect of FCC on HCC cell lines.

In the present study, the effect of FCC on proliferation and apoptosis of HCC cell line SMMC-7721 were investigated. In addition, to further investigate the molecular mechanisms of FCC on SMMC-7721 cells, we also studied the expression levels of proliferation marker PCNA and the apoptosis related proteins Bax and Bcl-2 by western blotting with FCC treatment.

## Results

### Effect of FCC on cell viability of SMMC-7721 cells

Chemical structure of FCC (MW = 192) was shown in Figure 1A. The compound, is the derivative of 3-formylchromone, formed when the hydrogen of the sixth carbon atom have been replaced with fluorine. In order to determine the effects of FCC on HCC, human HCC cell line SMMC-7721 was treated by FCC with different doses for 24 h (Figure 1B). The proliferation of SMMC-7721 cells was inhibited by FCC in a dose-dependent manner. Further experiments showed that FCC treatment inhibited the proliferation of SMMC-7721 cells in a time-dependent manner (Figure 1B).

**Figure 1:** **FCC Inhibited Cell Proliferation of SMMC-7721 cells. (A)** Chemical Structure of FCC. **(B)** Viability of SMMC-7721 cells treated with FCC. MTT assay was performed to measure cell growth inhibition rate at 24 h, 48 h and 72 h after FCC treatment. Data shown were representatives of three experiments.

### Effects of FCC on cell cycle and apoptosis of SMMC-7721 cells

The effect of FCC on cell cycle and apoptosis was observed with flow cytometry. SMMC-7721 cells were treated by FCC with various concentrations for 48 h. SMMC-7721 cells exhibited increased cell percentages in G0/G1 phase (Table 1) with an increase from 63.80% to 85.30%. The percentages of apoptotic cells were significantly increased in the treated group compared to control group (p < 0.05) (Table 1) in a dose-dependent manner. The apoptotic cells increased from a total of 2.8% to 48.2% for SMMC-7721 cells. Taken together, FCC treatment could induce HCC cell apoptosis and G0/G1 phase arrest.

**Table 1:** Effects of FCC on cell cycle and apoptosis of SMMC-7721 cells

**FCC (μg/mL)**	**G**_**0**_**/G**_**1**_	**S**	**G**_**2**_**/M**	**Apoptosis (%)**
0	63.8 ± 2.8	20.9 ± 3.8	15.3 ± 2.1	2.8 ± 1.3
2	69.1 ± 2.1	16.8 ± 2.4**	14.1 ± 1.8	9.5 ± 1.1**
5	76.4 ± 3.1	13.2 ± 1.4**	10.4 ± 0.9*	22.4 ± 1.9**
10	80.2 ± 1.9	11.0 ± 3.0**	8.8 ± 1.7**	37.5 ± 2.1**
20	85.3 ± 2.2	8.6 ± 2.3**	6.1 ± 2.0**	48.2 ± 1.7**

Cell cycle analysis and apoptosis of SMMC-7721 following FCC treatment for 48 h by flow cytometry. *p < 0.05, **p < 0.01, compared with control.

### Effects of FCC on PNCA, Bax and Bcl-2 expression

To further illustrate the molecular basis of the apoptosis induction by FCC, we investigated the effect of FCC on PCNA, Bax and Bcl-2 expression in SMMC. FCC significantly suppressed PCNA expression in a dose-dependent manner (Figure 2A and 2B). The total Bax expression level was increased with FCC treatment in a dose-dependent manner, while the total Bcl-2 expression level was decreased, resulting in a higher Bax/Bcl-2 ratio (Figure 2A and 2C).

**Figure 2:** **Effects of FCC treatment on PCNA, Bax, and Bcl-2 expression. (A)** SMMC-7721 cells were treated with FCC at doses of 0, 2, 5, 10 and 20 μg/ml for 48 h. The cell lysates were prepared and analyzed for PCNA, Bax and Bcl-2 expression by Western blot analysis. Equal loading was confirmed by stripping immunoblots and reprobing for β-actin. Data shown were representatives of three experiments. **(B)** Statistical analysis of PCNA quantification. **(C)** The ratio of Bax to Bcl-2 protein. *p < 0.05, **p < 0.01, compared with control.

## Discussion

To our knowledge, this is the first report describing the anti-tumor effect of FCC on HCC cell line SMMC-7721. Our data demonstrated that FCC could inhibit the proliferation of SMMC-7721 cells in vitro. It could down-regulate PCNA and Bcl-2 expression and up-regulate Bax expression. The results indicated that FCC could be developed as a novel anti-tumor agent for treating HCC.

The imbalance between cell proliferation and death is considered to be an important event in cancer progression [19,20]. Among the effects of anti-tumor reagents, apoptosis and growth inhibition are the most common responses on cancer cells [21,22]. In the present study, we observed that the viability of SMMC-7721 cells could be significantly decreased by FCC treatment for 24 h at various concentrations (ranging from 2 to 20 μg/ml) according to the MTT assay. The proliferation inhibition effect of FCC on SMMC-7721 cells in vitro is consistent with previous studies with other 3-formylchromone derivatives [13-15]. It is suggested that the potential of FCC treatment on the proliferation of human cancer cells in vitro.

Cell cycle regulation is one of the most important bioprocesses. Traditionally, the cell cycle is divided into four phases of G_1_-S-G_2_-M. DNA replication occurs during S phase, and chromosome segregation occurs during M phase. The S and M phases are separated by the so-called gap phases, G1 (before DNA replication) and G2 (before mitosis) [23]. It has been generally accepted that induction of cell cycle arrest and apoptosis are the important bio-reactions to anti-tumor reagents [24-26]. FCM cell cycle analysis in this study confirmed that FCC could induce a cell cycle arrest in G0/G1 phase, even the apoptosis when the damage couldn’t be repaired on time. PCNA is a protein which is the compound of cyclin D and cyclin-dependent kinases, involved in the proliferation cells, and it is specifically expressed in proliferating cell nuclei [27]. It has been shown that the levels of PCNA expression are higher in cancer tissues, including gastric, lung and breast cancer [28-30]. Several studies have emphasized the association of PCNA with tumor malignancy grade and prognostic significance in a number of malignancies [31,32]. Furthermore, it is reported that non-steroidal anti-inflammatory drugs (NSAIDs) could effectively postpone or hinder lung carcinogenesis through down-regulating PCNA expression in rat model [33]. Our results demonstrated that FCC could inhibit PCNA expression in SMMC-7721 cells with a dose-dependent manner. Therefore, the proliferation inhibition in SMMC-7721 cells by FCC might be ascribed to the suppressive effect on PCNA expression.

Members of the Bcl-2 family have been identified as key regulators of apoptosis including two opposing subfamilies [34]. Bcl-2 proteins often form heterodimer complexes with Bax proteins, which result in the release of cytochrome c from the mitochondria and subsequent induction of cell death [35]. Therefore, an increase in the ratio of Bax/Bcl-2 is considered as one of the major markers of pre-apoptosis. Several anti-tumor reagents have been confirmed to inhibit tumor growth by influencing the Bax/Bcl-2 ratio [36,37]. In the present study, our results also suggest that FCC effectively induces apoptosis in SMMC-7721 cells through up-regulation of the Bax/Bcl-2 ratio.

Taken together, our results suggested that FCC could induce G0/G1 cell cycle arrest and apoptosis in SMMC-7721 cells through suppressing PCNA expression and increasing Bax/Bcl-2 ratio, which advances our understanding on the molecular mechanisms of FCC in hepatocarcinoma management. However, the effects of FCC on SMMC-7721 were not investigated in animal models. More extensive research involving animal studies are needed in the future.

## Conclusions

FCC could significantly inhibit HCC cell growth in vitro through cell cycle arrest and inducing apoptosis by suppressing PCNA expression and modulating the Bax/Bcl-2 ratio.

## Methods

### Cell culture

Human HCC cell line SMMC-7721 was purchased from Cell Bank, Chinese Academy of Sciences (Shanghai, China). Cells were maintained in RPMI1640 medium (Gibco, Grand Island, NY) supplemented with 10% heatinactivated fetal bovine serum (Gibco, Grand Island, NY) at 37°C in a humidified atmosphere containing 5% CO_2_. In order to inhibit aminoxidase, aminoguanidine was added into RPMI1640 medium at a final concentration of 1 mmol/L.

All studies have been approved by The Ethics Committee of Changhai Hospital and performed in accordance with the ethical standards.

### Antibodies and reagents

Antibodies against PCNA, Bax and Bcl-2 were purchased from Santa Cruz (Santa Cruz Biotechnology, Santa Cruz, CA, USA). FCC, trypsin and MTT were obtained from sigma (Sigma, St. Louis, MO, USA). Cell Cycle Detection Kit was purchased from Thermo (Thermo Fisher Scientific Inc, NH, USA).

### Cell viability assay

The effect of FCC on cell viability was measured by 3-(4, 5-dimethylthiazol-2-yl)-2, 5-diphenyl tetrazoliumbromide (MTT) assay. The cells were plated at a density of 1 × 10^4^ per well in 96-well plates overnight and then treated by FCC with different concentrations of cell solution (0, 2, 5, 10, and 20 μg/ml). After incubation for 24 h, 48 h and 72 h at 37°C in a humidified incubator, MTT (5 mg/ml in phosphate buffered saline (PBS)) was added to each well and incubated for 4 h; then the medium was totally removed, 0.15 ml of buffered DMSO was added to each well. The absorbance was recorded on a microplate reader at the wavelength of 490 nm. The effect on cell proliferation was assessed as the percent cell viability wherein vehicle-treated cells were taken as 100% viable.

### Cell cycle analysis

After FCC treatment, the DNA content and cell cycle distribution of SMMC-7721 cells were determined by flow cytometry. Cells plated at a density of 1 × 10^6^ per well in 6-well plates, treated with FCC and then harvested at 24 h. The cells were washed twice with PBS. They were then fixed in cold 70% ethanol and stored at 4°C for 30 min. Then ethanol was removed and the cells were resuspended in PBS. The fixed cells were then washed with PBS, treated with RNase (100 mg/ml), and stained with Propidium Iodide (PI, 50 mg/ml) in the dark for 30 min at 37°C. Cell cycle was analyzed by flow cytometry.

### Western blot analysis

SMMC-7721 cells were treated with FCC (0, 2, 5, 10, and 20 μg/ml) for 48 h in complete cell medium. After 48 h of treatment, cells were harvested and cell lysates were prepared and stored at -80°C for later use. The protein content in the lysates was determined using a modified Lowry assay [38]. For Western blot analysis, 50 μg of protein from each sample were subjected to separate on a SDS-PAGE gel. After electrophoresis, proteins were electroblotted to polyvinylidene difluoride (PVDF) membranes, and subsequently incubated in blocking buffer (5% nonfat dry milk) for 12 h at 4°C. The blots were incubated with appropriate primary antibody, washed, and incubated with horseradish peroxidase (HRP)-conjugated secondary antibody. The blots were detected with chemiluminescence.

### Statistical analysis

All data represents at least three independent experiments and results were shown as mean ± SD. Statistical differences between two groups were determined by Student’s *t*-test. A significant difference was considered as p < 0.05.

## Abbreviations

HCC: Hepatocellular carcinoma; FCC: 6-fluoro-3-formylchromone; NSAIDs: Non-steroidal anti-inflammatory drugs; MTT: 3-(4, 5-dimethylthiazol-2-yl)-2, 5-diphenyl tetrazoliumbromide; PBS: Phosphate buffered saline; PVDF: Polyvinylidene difluoride; HRP: Horseradish peroxidase.

## Competing interests

The authors declare that they have no competing interests.

## Authors’ contributions

YZ and KZ designed this study. JW performed the statistical analysis. CS and GJ carried out the study. YZ collected important background information, XZ and TH drafted the manuscript. All authors read and approved the final manuscript.

## Pre-publication history

The pre-publication history for this paper can be accessed here:

http://www.biomedcentral.com/1471-230X/14/62/prepub
